# Systemic Administration of Neutral Electrolyzed Saline as a Novel Treatment for Rheumatoid Arthritis Reduces Mechanical and Inflammatory Damage to the Joints: Preclinical Evaluation in Mice

**DOI:** 10.1155/2022/1717614

**Published:** 2022-06-02

**Authors:** Sergio A Zaizar-Fregoso, Brenda A Paz-Michel, Alejandrina Rodriguez-Hernandez, Juan Paz-Garcia, Nomely S. Aurelien-Cabezas, Daniel Tiburcio-Jimenez, Valery Melnikov, Efren Murillo-Zamora, Osiris G Delgado-Enciso, Ariana Cabrera-Licona, José Guzman-Esquivel, Carlos E Barajas-Saucedo, Iram P Rodriguez-Sanchez, Margarita L Martinez-Fierro, Norma A Moy-López, Agustin Lara-Esqueda, Jorge Guzman-Muñiz, Marina Delgado-Machuca, Ivan Delgado-Enciso

**Affiliations:** ^1^Facultad de Medicina, Facultad de Psicologia, Universidad de Colima, Colima 28040, Mexico; ^2^Instituto Estatal de Cancerología, Servicios de Salud del Estado de Colima, Colima 28085, Mexico; ^3^Esteripharma SA de CV, Atlacomulco 50450, Estado de Mexico, Mexico; ^4^Centro Hospitalario Unión, Villa de Álvarez 28970, Colima, Mexico; ^5^Instituto Mexicano Del Seguro Social, Villa de Alvarez 28983, Colima, Mexico; ^6^Universidad Autonoma de Nuevo Leon, Facultad de Ciencias Biologicas, San Nicolás de los Garza 66455, Nuevo Leon, Mexico; ^7^Unidad de Medicina Humana y Ciencias de La Salud, Universidad Autonoma de Zacatecas, Zacatecas 98160, Mexico; ^8^Facultad de Psicologia y Terapia de la Comunicación Humana, Universidad Juarez del Estado de Durango, Durango 34120, Mexico

## Abstract

Rheumatoid arthritis is globally present in about 1% of the population. This autoinflammatory disease modifies the connective tissue, causing pain and inflammation of the joints. Over time, it causes the loss of joint cartilage and bone mass, decreasing the patient's quality of life. Treatment options now available either give symptomatic alleviation or alter the disease process. Nonetheless, adherence to chronic treatment is typically limited due to adverse effects. As a result, new therapy approaches, such as systemic administration of neutral electrolyzed saline to improve patients' quality of life, are being investigated. The study is a randomized prospective preclinical trial with a single-blind and a 4-arm parallel group using a collagen-induced mice model to generate rheumatoid arthritis. It was carried out on 36 male BALB/c mice, with the primary outcome measure being a scoring system for histopathologic assessment. When all groups are compared, there are significant differences. In addition, the animal model was validated by the healthy group. The animals treated with neutral electrolyzed saline had much less cartilage degradation, bone erosion, pannus development, and inflammation than the placebo-treated mice. Serum IL-6 levels were evaluated in parallel with disease severity expressed as synovitis grading of the affected joints. Spearman's rank correlation coefficient (Rs) = 0.399 (*P*=0.016) between serum IL-6 levels and the synovitis grading suggests a direct correlation between IL-6 production and disease severity. An additional trial of 20 male BALB/c mice (10 treated with placebo and 10 with neutral electrolyzed saline for 30 days) showed no clinical nor histopathological evidence of adverse effects. According to histopathological and blood test results, we conclude that neutral electrolyzed saline minimizes mechanical and inflammatory damage to the joint and may be helpful as an alternative to rheumatoid arthritis therapy.

## 1. Introduction

Rheumatoid arthritis (RA) is an autoimmune disorder that targets the connective tissue [1], ultimately leading to the destruction of joints, which causes the patient's functional decline, disability, pain, and swelling [2]. It affects mainly women, although it is estimated that 1% of the world's population suffers from it [3], with pain as the most common symptom [4].

Approved RA treatments include NSAIDs, DMARDs, corticosteroids, methotrexate, TNF-blocking, interleukin blocking, B-cell depletion, and CTLA4-Ig [5–9]; they either give clinical relief or change the disease process [10]. Unfortunately, most of them are ineffective, and side effects typically restrict their chronic use [11].

Therefore, there is an opportunity to explore new treatment options, which is the objective of this study by evaluating histopathological and functional changes in a murine RA model, treated or not with neutral electrolyzed saline. This solution has been activated by a controlled electrochemical process that leads to reactive chlorine and oxygen species (ROS) formation from a sodium chloride saline solution [12].

Evidence about ROS intervention during RA is controversial. On the one hand, it leads to tissue damage, while on the other hand, it mediates disease severity by reducing tissue damage [12, 13]. In addition, some studies about treatments with NES rich in ROS have shown a crucial anti-inflammatory effect [14]. The induction of damage or a beneficial effect depends on ROS concentration in the NES.

Murine arthritis models are highly accepted, particularly the collagen-induced arthritis (CIA) mouse model [15]. It is recognized in preclinical treatment models because they share clinical, histological, and immunological characteristics with human RA [16].

## 2. Materials and Methods

The study consisted of two stages. First, the safety and toxicity of parenteral administration (intraperitoneal injection) of neutral electrolyzed saline in mice fed a high-fat diet were analyzed. In a second stage, the therapeutic effect of the neutral electrolyzed saline (intraperitoneal injection) was evaluated in an animal model of rheumatoid arthritis.

### 2.1. Neutral Electrolyzed Saline

Neutral electrolyzed saline is an aqueous saline solution of sodium chloride, activated by a controlled electrolysis process (patent no. MX330845 B), and thus resembles activated saline, electrolyzed saline, or electrolyzed water. It had a neutral pH (6.0–7.5), and its active ingredient was 0.002% of active species of chlorine and oxygen [17]. The parenteral electrolyzed saline, HOMEOSTECH® (provided by Esteripharma SA de CV, Mexico City, Mexico, as an experimental, not commercial product), and sterile injectable items used in this therapy comply with good manufacturing practices (GMP).

### 2.2. Ethics

This experimental procedure was approved by the Research and Ethics Committee of the Instituto Estatal de Cancerologia, Secretaria de Salud del Estado de Colima (Colima, Mexico). The experimental subjects were handled in accordance with institutional procedures and satisfied the Mexican legislation related to laboratory animal practice (NOM-062-ZOO-1999) and the National Academy of Sciences Guide for the Care and Use of Laboratory Animals (2011). In addition, all animals were sacrificed following the American Veterinary Medical Association's 2013 criteria for animal sacrifice.

### 2.3. In Vivo Toxicity of Neutral Electrolyzed Saline

Male BALB/c mice between 8 and 12 weeks of age with an average weight of 24–30 g (Envigo, Huntingdon, UK) were included, and they were fed a high-fat diet (Western diet) as previously described [18]. All animals were kept at 21°C ± 2°C in a 12-hour light-dark cycle with free food and water intake. Using random allocation software, twenty mice were randomized into two parallel groups of 10 animals each.

For this assay, two groups were formed. Group 1 (*n* = 10) was injected parenterally (intraperitoneally) with physiological saline solution (0.9% of NaCl) (placebo group) at a dose of 40 *µ*L/d for 30 consecutive days. Group 2 (*n* = 10) was injected intraperitoneally with neutral electrolyzed saline (NES group) at a dose of 40 *µ*L/d for 30 consecutive days.

The weight of the mice was quantified once a week prior to parenteral injection. Weight was expressed in grams. Mice were observed daily by a single examiner to assess for clinical signs of toxicity. Some of the clinical observations of the Irwin test and functional observational battery (FOB) were considered: autonomic evaluation (piloerection, diarrhea, and breathing), neuromuscular evaluation (seizures, posture, and gait), and behavioral evaluation (aggressiveness, sedation, and stereotypy) [19]. After the treatment period, all animals were euthanized by decapitation. The livers and kidneys were dissected and morphologically analyzed.

### 2.4. Study Design for Rheumatoid Arthritis Treatment with Neutral Electrolyzed Saline

According to the “ARRIVE Essential 10” guidelines for Animal Research [20], the study was carried out as a randomized prospective preclinical trial with a single-blind and a 4-arm parallel group (see Figure 1).

### 2.5. Murine Arthritis Model

The model includes two phases: induction and development of the disease. The induction starts with the immunization and lasts until the development phase is observed, detecting any visible sign of the disease. In this case, the development phase started on day 33, from the first immunization, when mechanical allodynia was observed. Then, immunization emulsion and boost emulsion were prepared as previously described by Raza et al. [21].

### 2.6. Sample Size

The sample size was calculated by the resource equation [22] and resulted in 36 subjects. However, since the literature reported a 50% success rate in the induction phase of RA [11], 72 subjects were included and induced.

### 2.7. Animals, Inclusion Criteria, and Randomization

Male BALB/c mice between 8 and 10 weeks of age were included and weighed 25–28g (Envigo, Huntingdon, UK). For the animals selected to develop collagen-induced arthritis, the first sign of clinical disease (allodynia) occurred on day 33 from the first immunization; a whole sample of 27 mice was randomized into three parallel groups of nine animals each, using a random allocation software package [23]. The fourth group of 9 untreated mice (the healthy group) was randomly confirmed at the beginning of the experiment, before the induction of the AR disease in the remaining mice. Animals which were induced but developed no clinical manifestations of the disease at day 33 were excluded. Elimination criteria included dead subjects during the study period without replacement or any subject that developed any other type of illness. All animals were kept at 21°C ± 2°C in a 12-hour light-dark cycle with free food and water intake.

### 2.8. Intervention

According to their corresponding group, all the animals (except healthy individuals) began the treatment in the development phase. The healthy group (not induced into AR) received no treatment, and the placebo group received an intraperitoneally physiological saline solution. According to their group, the two remaining groups received 20 *μ*L/d or 40 *μ*L/d of neutral electrolyzed saline intraperitoneally.

All animals were euthanized by decapitation following the protocols outlined above and after the treatment period. Blood samples were obtained afterward, and the serum was separated and analyzed for inflammatory mediator interleukin-6 (IL-6) levels. According to the manufacturer's instructions, the analysis was made using the mouse IL-6 ELISA Kit RAB0308 (Sigma-Aldrich, Saint Louis, MO, USA) and performed in triplicate. Simultaneously, a dissection of the left knee was conducted for histological processing.

### 2.9. Histological Processing

All tissues initially analyzed were preserved in 10% buffered formalin and embedded in paraffin. For histopathologic evaluation, 5 *μ*m slices were stained with hematoxylin and eosin. Only the kidney sections were stained with Masson's trichrome. Images were taken with an Axiocam MRC-5 model digital camera (Zeiss GmbH, Jena, Germany) mounted on an AxioPlan 2M model bright-field optical microscope (Zeiss GmbH) with a motorized stage, and A-plan x4, x10, x20, and x40 objectives were used to grade the slices. All the photographs were acquired under the same lighting and exposure conditions. AxioVision software version 4.0 was used to conduct the analyses (Zeiss GmbH, Jena, Germany).

### 2.10. Histological Assessment

Toxicity animal model: for kidney damage detection, the main parameters evaluated were acute tubular necrosis, tubular atrophy, tubulointerstitial fibrosis, and interstitial infiltrate of inflammatory cells. In addition, all renal histological findings were evaluated and quantified as a percentage of the cortical area affected by each defined parameter. x20 and x40 objectives were used to evaluate kidney slices.

For liver damage detection, the main parameters evaluated were the number of hepatocytes, inflammatory cells, hepatic ballooning, and cell binucleation; all findings were evaluated under 400x magnification field, as the percentages of steatohepatitis and necrosis, previously reported.

Rheumatoid arthritis animal model: mice's knee joints were evaluated microscopically using a modified scoring method for inflammation, cartilage injury, pannus development, bone resorption, and ectopic chondrocytes on a scale of 0 to 3. This score was determined by two blinded observers using a modified version of the previously published mouse scoring method of Tseng et al. [24], where 0 indicates normal, 1 represents minor damage or less than 50% of the variable being assessed, and 2 means substantial damage or more than 50% of the variable being tested. In addition, we added the synovitis classification score by summing the scores of excess tissue formation (hyperplasia), pannus formation, and inflammation [25, 26].

### 2.11. Statistical Analysis

Statistical tests were conducted with IBM SPSS version 20 software (IBM SPSS, Chicago, Illinois, USA) with a statistical significance level of *p* < 0.05. Since the Shapiro–Wilk test indicated nonnormal data distribution, all variables are shown with medians and the 25th and 75th percentiles (Q1 and Q3). The Kruskal–Wallis test was used to compare groups, with the Mann–Whitney *U*-test used as a post hoc analysis. Finally, Spearman's test was used to calculate correlations.

## 3. Results

### 3.1. In Vivo Toxicity Model

During the study, there was no evidence of toxic effects clinically detected in mice, according to FOB analysis. The mice did not present autonomic alterations (piloerection, diarrhea, and abnormal breathing), neuromuscular alterations (seizures, abnormal posture, and abnormal gait), or behavioral alterations (aggressiveness, sedation, and stereotypy) (data not shown). In addition, no animal mortality was reported during the administration of NES. The weight of the mice did not show any differences when comparing the two groups (Table 1).

Kidney and liver weight did not differ between groups (Table 2). The animals injected with NES or physiologic saline solution did not present interstitial fibrosis, tubular atrophy, or acute tubular necrosis at the renal histological level. In addition, the interstitial infiltrate of inflammatory cells was similar when comparing both groups (Table 2).

It is essential to mention that the mice were fed a high-fat diet, simulating individuals on a Western diet. This is relevant to consider when analyzing the liver histological data mentioned in Table 1. Animals treated with NES presented with a significant increase in regenerative histological markers (higher number of hepatocytes, binucleation) as well as significantly fewer histological damage markers (steatohepatitis, necrosis, and hepatic ballooning) when compared with the placebo group (physiologic saline solution). However, the number of inflammatory cells in the liver tissue was similar in both groups (Table 2).

### 3.2. Murine Arthritis model

All the mice included in the treatment and follow-up concluded the study and were analyzed (36 individuals, 9 mice per group).  Table 3 shows the histopathological evaluations of joints and an intergroup comparison, and Table 4 shows the results of the post hoc analysis.

Significant differences were found when comparing all groups. The healthy group had significantly less joint damage than all other groups, confirming the animal model (Table 4). Treatment with neutral electrolyzed saline, at both doses, significantly reduced cartilage damage, bone erosion, pannus formation, and inflammation compared with the placebo group (Table 4). The experimental treatment did not produce changes in excess tissue formation or the presence of ectopic chondrocytes since no significant differences were found between groups treated with both doses of neutral electrolyzed saline (Table 4). However, a more conserved joint was observed in the group treated with the highest dose (Figure 2). The beneficial effects of the treatment are evident in Figure 2.

All histopathological scored variables have a high positive correlation, showing a direct relationship between the studied morphological alterations (Table 5).

Serum level values of the inflammatory mediator IL-6 were 5.1 pg/mL (*Q*1 = 4.9 to *Q*3 = 7.8), 13.9 pg/mL (*Q*1 = 6.0 to *Q*3 = 20.1), and 6.4 pg/mL (*Q*1 = 5.5 to *Q*3 = 10.1) in the healthy, NES20, and NES40 groups, respectively. The Kruskal–Wallis test shows a significant difference between the groups (*P* < 0.001). The post hoc analysis (Mann–Whitney *U*-test) shows that the NES20 group has elevated IL-6 levels in comparison with the healthy (*P* < 0.001) and NES40 (*P*=0.026) groups, while the IL-6 levels from the NES40 and healthy groups were not significantly different (*P*=0.116). To establish possible correlations between IL-6 levels and the severity of arthritis, serum IL-6 levels were evaluated in parallel with disease severity expressed as synovitis grading of the affected joints. The Spearman correlation coefficient (Rs) = 0.399 (*P*=0.016) between serum IL-6 levels and the synovitis grading suggested a direct correlation between IL-6 production and disease severity.

## 4. Discussion

Parenteral administration of neutral electrolyzed saline (NES) was safe and reduced inflammation and other joint degenerative changes caused by induced rheumatoid arthritis in a mouse model. In addition, the administration of NES at the highest dose prevented the elevation of IL-6 levels. Most benefits were linked to administering the highest dose (40 *μ*L vs. 20 *μ*L per day), suggesting a dose-response relationship.

Chronic articular inflammation causes the synovium to enlarge, resulting in an aberrant pannus, invading and destroying local articular structures [27]. Due to the highly similar composition of the ROS generated by the immune system and those included in the neutral electrolyzed saline as active species, the NES induces an immunomodulatory effect in the organism that reduces the systemic inflammatory process, as was recently demonstrated in a clinical trial of patients with COVID-19 (Delgado-Enciso et al., 2021). Hence, we hypothesize that a similar effect is responsible for the observed results, where the parenteral injection of NES decreases inflammation and joint degeneration in an animal model of RA (see Figure 2).

In addition, the beneficial effects of NES administration are reflected in the modulation of the IL-6 levels in the animal model of RA. The group that received the highest dose of NES (40 *μ*L/day) showed no difference in their IL-6 levels compared with the healthy group, while the values of the group that only received 20 *μ*L/day were significantly elevated compared with the healthy or NES40 groups. Besides, a significant correlation was found between serum IL-6 levels and the synovitis grading, suggesting a direct correlation between IL-6 production and disease severity. Interleukin-6 (IL-6) is overproduced in the joints of patients with rheumatoid arthritis, suggesting that IL-6 production is a crucial factor in the pathogenesis of the disease [27, 28].

It has been previously postulated that blocking or inhibiting IL-6 is a valuable strategy for treating RA since there is a clear association between IL-6 levels and the quality of life in RA patients [27, 28]. In that sense, and according to the findings in the animal model of this study, the administration of NES was beneficial in modulating IL-6 levels, which correlated with a reduction in joint damage, especially for the group treated with the highest dose of NES (NES40). Furthermore, a recent in vitro report showed that hypochlorous acid (HOCl), one of the main components of NES, is capable of interacting with IL-6, blocking or reducing interaction with its receptors in a dose-dependent manner [29], although more studies are needed in this regard.

As was previously mentioned, there are several treatments for RA. However, their useful life is limited by the side effects they produce. In this study, NES showed no side effects that may limit its application as an alternative treatment, potentially providing the patient with all the beneficial effects observed in this study (see Tables 2 and 3), which could be even better than those related to current therapies. For example, while glucocorticoids, NSAIDs, and DMARDs do not prevent bone loss in RA, neutral electrolyzed saline is probed to preserve the bone structure close to natural (see Figure 2). This is clear evidence of the significant therapeutic potential that NES could offer to RA patients.

An in vivo toxicity model showed that parenteral administration of NES for 30 days did not generate any adverse effects and was well tolerated. Clinical observations (Irwin test and functional observational battery) were normal throughout the follow-up. In addition, no adverse alterations were found in the liver or kidney tissues (Table 2). The animal model used in the toxicity test had a western diet rich in fat, consistent with the development of steatohepatitis and other associated histological changes. In this sense, the administration of NES reduced the percentage of liver tissue with steatohepatitis, necrosis, and hepatic ballooning. These changes caused by the NES administration can be considered beneficial and should be analyzed in further research. Furthermore, the safety of parenteral administration of NES (intravenously) has been demonstrated in a recent clinical trial that showed benefits in patients with COVID-19 [17, 30]. In that trial, no serious adverse effects were observed, and it was generally well tolerated by patients [17].

The current study has certain flaws. The trial did not include current therapy, such as NSAIDs or DMARDs. In this regard, the aim of this study was just to determine the efficacy of the neutral electrolyzed saline on RA and not to make a comparison of efficacy among treatments. A gold standard therapy must be included once the efficacy of NES is evaluated in clinical models [30].

## 5. Conclusions

Rheumatoid arthritis treatment with neutral electrolyzed saline reduces the joint's mechanical and inflammatory damage, which is correlated with a reduction in IL-6 serum levels.

## Figures and Tables

**Figure 1:** Schematic representation of the study in the rheumatoid arthritis mouse model. After the induction of the pathology (collagen-induced arthritis (CIA) model), the animals were randomized into three groups, one with a placebo and the others with the administration of 20*µ*l (NES20) or 40 *µ*l (NES40) of neutral electrolyzed saline, all of them daily. An additional group remained without disease induction (healthy) or treatment. After 30 days of treatment and follow-up, the animals were sacrificed for histopathological analysis of their joint disease. Blood samples were also taken for IL-6 analysis.

**Figure 2:** Histology images of the knee joints from the four groups, stained with hematoxylin and eosin. One joint per group, randomly selected, is shown at 10X. All of the photographs were acquired with the same microscope and under the same lighting and exposure conditions. The red arrows indicate articular cartilage, observed intact in the healthy group. In contrast, the placebo group has an irregular thickening and significant bone erosion, and there is evidence of joint fusion (black arrow) with pannus formation. In group NES20, the thickness of the articular surface is conserved (red arrow) with isolated foci of erosion (black arrow). The representative joint from group NES40 shows remarkably conserved thickness without erosion data.

**Table 1:** Intergroup analysis of weight variations.

Parameter	Placebo	NES	*P* value^†^
	Median (Q1–Q3), *N* = 10 in each group		
Week 1	25.37 (24.85–29.65)	23.82 (22.27–29.31)	0.082
Week 2	24.76 (23.96–30.29)	24.06 (22.33–29.47)	0.199
Week 3	24.95 (24.46–30.94)	24.37 (23.19–29.29)	0.186
Week 4	26.99 (25.78–29.11)	24.34 (23.63–29.10)	0.082

NES : neutral electrolyzed saline; Q1 and Q3: 25th and 75th percentiles. ^*∗*^Weight is expressed in grams. ^†^Mann–Whitney *U*-test. .Statistical significance: *P* < 0.05. Two-tailed *P* values are shown.

**Table 2:** Intergroup comparison of renal and hepatic histological findings.

Parameter	Placebo, median (Q1–Q3), *N* = 10 in each group	NES	*P* value^†^
Renal histological findings^*∗*^			

Tubular necrosis (%) Tubular atrophy (%) Interstitial infiltrate inflammatory cells (%) Tubulointerstitial fibrosis (%)	0.0 (0.0–0.0) 0.0 (0.0–0.0) 5.0 (5.0–10.0) 0.0 (0.0–0.0)	0.0 (0.0–0.0) 0.0 (0.0–0.0) 0.0 (5.0–5.0) 0.0 (0.0–0.0)	1.000 1.000 0.089 1.000

Liver histological findings^^*∗∗*^^			

Hepatocytes (*n*) Inflammatory cells (*n*) Steatohepatitis (%) Necrosis (%) Hepatic ballooning (*n*) Hepatic binucleation (*n*)	59.5 (41.7–77.2) 45.0 (40.0–51.2) 75.0 (65.0–87.5) 47.5 (34.4–60.0) 11.0 (1.7–19.0) 6.0 (3.7–9.0)	69.5 (46.7–82.7) 46.0 (41.0–55.2) 55.0 (37.5–70.0) 35.0 (22.5–50.0) 0.0 (0.0–4.0) 7.0 (4.0–10.2)	0.028 0.369 0.001 0.001 0.001 0.029

Organ weight^*∗∗∗*^			

Right kidney Left kidney Liver	0.23 (0.17–0.25) 0.22 (0.15–0.26) 1.58 (1.49–1.76)	0.15 (0.14–0.25) 0.15 (0.14–0.26) 1.23 (1.21–1.79)	0.404 0.343 0.226

NES : neutral electrolyzed saline; Q1 and Q3: 25th and 75th percentiles.^∗^Percentage of findings in the renal cortex. ^*∗∗*^Per histological field 40x. ^*∗∗∗*^Weight expressed in grams. ^†^Mann–Whitney *U*-test. Statistical significance: *P* < 0.05. Two-tailed *P* values are shown.

**Table 3:** Histopathological intergroup analysis.

Histopathological scores^*∗*^	*N* = 9 in each group				
	Healthy	Placebo	NES20	NES40	*P* value^†^
		Median (Q1–Q3)			
Cartilage damage	0 (0–0)	2 (2–3)	2 (1–2)	1 (1–1)	<0.001
Bone erosion	0 (0–0)	3 (3–3)	1 (1–3)	1 (1–2)	<0.001
Excess tissue formation	0 (0–0)	2 (2–3)	2 (2–2)	1 (1–2)	<0.001
Pannus formation	0 (0–0)	3 (2–3)	1 (1–2)	2 (1–2)	<0.001
Ectopic chondrocytes	0 (0–0)	2 (2–3)	1 (0–3)	2 (2–3)	<0.001
Inflammation	0 (0–0)	2 (2–3)	2 (1–2)	1 (1–1)	<0.001
Synovitis grading^^*∗∗*^^	0 (0–0)	8 (6–8)	5 (3–6)	4 (3–5)	<0.001

NES : neutral electrolyzed saline 20 (20 *µ*l/d) or 40 (40 *µ*l/d); Q1 and Q3: 25th and 75th percentiles. ^*∗*^Scoring system by Tseng H–W et al. (2016); ^†^Kruskal–Wallis test; ^*∗∗*^histopathological synovitis score by Krenn et al. (2002)

**Table 4:** Pairwise comparison of histopathological scores with the Mann–Whitney *U*-test.

Histopathological scores^*∗*^	H vs. NES20	H vs. NES40	H vs. P	P vs. NES20	P vs. NES40	NES20 vs. NES40
Cartilage damage	0.011	0.004	0.007	0.046	0.046	0.234
Bone erosion	0.015	0.006	0.005	0.033	0.006	0.748
Excess tissue formation	0.008	0.007	0.007	0.257	0.157	0.763
Pannus formation	0.016	0.007	0.006	0.008	0.020	0.336
Ectopic chondrocytes	0.023	0.007	0.006	0.068	0.480	0.260
Inflammation	0.006	0.004	0.006	0.034	0.010	0.058
Synovitis grading^*∗∗*^	0.007	0.007	0.007	0.020	0.011	0.678

H: healthy group; *p*: placebo group (physiological saline solution); NES 20 : neutral electrolyzed saline 20 *µ*l/d; NES 40 : neutral electrolyzed saline 40 *µ*l/d. ^*∗*^Scoring system by Tseng H–W et al. (2016); ^*∗∗*^histopathological synovitis score by Krenn et al. (2002). *p* Two-tailed *p* values are shown.

**Table 5:** Spearman's correlation coefficients between the histopathological scores of all groups.

Histopathological Scores	Cd	Be	Etf	*P*f	Ec	I	Sg
Cartilage damage (Cd)	1.000						
Bone erosion (Be)	0.782^*∗*^	1.000					
Excess tissue formation (Etf)	0.890^*∗*^^*∗*^	0.678^*∗*^	1.000				
Pannus formation (Pf)	0.826^*∗*^	0.848^*∗*^	0.850^*∗*^	1.000			
Ectopic chondrocytes (Ec)	0.747^*∗*^	0.742^*∗*^	0.700^*∗*^	0.859^*∗*^	1.000		
Inflammation (I)	0.814^*∗*^	0.785^*∗*^	0.764^*∗*^	0.824^*∗*^	0.703^*∗*^	1.000	
Synovitis grading (Sg)	0.896^*∗*^	0.810^*∗*^	0.925^*∗*^	0.958^*∗*^	0.812^*∗*^	0.905^*∗*^	1.000

^*∗*^Correlation is significant at the 0.01 level (2-tailed).

## Data Availability

The current study contains all the necessary data. The datasets used and analyzed during the current work are available from the corresponding author upon reasonable request.
